The article "Effects of Coculture Fibroblasts and Vascular Endothelial Cells on Proliferation and Osteogenesis of Adipose Stem Cells" was retracted in 2023. Reasons: unreliable results or conclusions; concerns about the data; concerns about the peer review; concerns about the citations.

# Effects of Coculture Fibroblasts and Vascular Endothelial Cells on Proliferation and Osteogenesis of Adipose Stem Cells

**DOI:** 10.1155/2022/6288695

**Published:** 2022-01-13

**Authors:** Xinyu Liao, Ruiying Zhong, Hong Zhang, Fuke Wang

**Affiliations:** ^1^Department of Sports Medicine, The First Affiliated Hospital of Kunming Medical University, Yunnan Province, China; ^2^Department of Psychiatry, The First Affiliated Hospital of Kunming Medical University, Kunming, 650032 Yunnan Province, China

## Abstract

**Background:**

The development of tissue engineering provides a new method for the clinical treatment of bone defects, but the problems of slow formation and slow vascularization of tissue engineered bone have always existed. Studies have shown that the combined culture system of vascular endothelial cells and adipose stem cells is superior to single cell in repairing bone defects. With the excellent proliferation ability, secretion of synthetic collagen and a variety of regulatory factors and fibroblasts can differentiate into osteoblasts and have the potential to be excellent seed cells involved in tissue engineering bone construction.

**Objective:**

To investigate the effects of combined culture of fibroblasts, vascular endothelial cells, and adipose stem cells on proliferation and osteogenic differentiation of adipose stem cells.

**Methods:**

The cells were divided into 4 groups: adipose stem cell group, adipose stem cell+vascular endothelial cell coculture group, adipose stem cell+fibroblast coculture group, and adipose stem cell+vascular endothelial cell+fibroblast coculture group. The morphological changes of the cells were observed under an inverted microscope. After 1, 3, 5, 7, and 9 days of coculture, the proliferation of adipose stem cells in each group was detected by a CCK-8 method and the growth curve was plotted. Adipose stem cells in each group were stained with alizarin red and alkaline phosphatase at days 7, 14, 21, and 28. At the third week of coculture, Western blot was used to detect the expression level of bone morphogenetic protein 2 of adipose stem cells in each group. *Results and Conclusions*. (1) After 14 days of culture, some cells in the adipose stem cell+vascular endothelial cell+fibroblast coculture group fused into clumps and distributed in nests, while the adipose stem cells in the adipose stem cell group had a single cell morphology and no cell clusters were observed. (2) The cell growth curves were basically the same in each group, and the absorbance value increased gradually. The absorbance value of the adipocyte+vascular endothelial cell+fibroblast coculture group was the highest, followed by the adipocyte+fibroblast coculture group and then the adipocyte+fibroblast coculture group. (3) Alizarin red staining showed negative reaction in each group on the 7th day, and a small number of red positive cells gradually appeared in each group as time went on. On the 28th day, red positive cells were found in all groups, and most of them were in the coculture group of adipose stem cells+vascular endothelial cells+fibroblasts, showing red focal. The coculture group of adipose stem cells+vascular endothelial cells and adipose stem cells+fibroblasts was less, and the adipose stem cell group was the least. On day 28 of alkaline phosphatase staining, cells in each group had red positive particles, and the adipose stem cell+vascular endothelial cell+fibroblast coculture group and adipose stem cell+fibroblast coculture group had the most, followed by the adipose stem cell+vascular endothelial cell coculture group and then the adipose stem cell group. (4) Bone morphogenetic protein 2 was expressed in all groups, especially in adipose stem cell+fibroblast coculture group and adipose stem cell+vascular endothelial cell+ fibroblast coculture group. (5) Fibroblast could promote adipose stem cell osteogenic differentiation better than vascular endothelial cells, but the proliferation effect was not as good as vascular endothelial cells. The coculture system of fibroblast combined with vascular endothelial cells and adipose stem cells promoted the proliferation of adipose stem cells and the rapid and efficient differentiation of adipose stem cells into osteoblasts.

## 1. Introduction

From the physiological point of view, the maintenance of bone tissue function is completed by the interaction, promotion, and joint action of various cells, extracellular matrix, and various cytokines. Previous experiments have confirmed that the combined culture system of vascular endothelial cells (VECs) and adipose-derived stem cells (ADSCs) has better ability to repair bone defects than single cells [1].

Fibroblasts (FB) and osteoblasts are derived from embryonic mesenchymal cells and maintain high proliferation characteristics, which can differentiate into osteoblasts under certain conditions and express osteogenic markers [2]. Fibroblasts exist in various tissues of the body and can be easily and quickly obtained. They can be autologous transplanted and can differentiate into three layers [3]. Fibroblast cytokines play a key role in the growth and development of skeletal system and fracture healing. Therefore, this study considers the application of fibroblasts in the combined culture system of adipose stem cells and vascular endothelial cells to study the effects of fibroblasts and vascular endothelial cells on proliferation and osteogenic differentiation of adipose stem cells. It provides experimental and theoretical basis for selecting seed cells for bone tissue engineering to promote rapid osteogenesis and vascularization of tissue-engineered bone and to explore the interaction between cells.

## 2. Experimental Materials

The main design of the experiment is in vitro cytological observation experiment, and the experiment was conducted at the Kunming Institute of Zoology, Chinese Academy of Sciences, from April 2019 to February 2020.

The experimental material starring includes the following three parts:

1. Cells and source: adipocytes were derived from Kunming Cell Bank, Committee of Typical Culture Treasures, Chinese Academy of Sciences (cell line number KCB2010101). Vascular endothelial cells were derived from Kunming Cell Bank, Committee of Typical Culture Treasures, Chinese Academy of Sciences (cell line number KCB2012087YJ). The fibroblasts were derived from Kunming Cell Bank, Committee of Typical Culture Treasures, Chinese Academy of Sciences (cell line number KCB2019021YJ).
2. Main reagents for the experiment: bone morphogenetic protein 2 (MCE, USA); CCK-8 (Gibco, USA); EDTA (Sigma); trypsin (Sigma); low sugar DMEM medium (Gibson); methyl cellulose (R&D Corporation); endothelial cell culture medium (ScienCell); Western Blot kit (Gibco, USA); dimethyl sulfoxide (Sigma); alizuhong (Shanghai Saieise Reagent Co., Ltd.); BCIP/NBT Alkaline Phosphatase Coloration Kit (Beyotime Biotechnology Institute); and hematoxylin (Beyotime Biotechnology Institute) are the main reagents.
3. Main instruments for the experiment: ultraclean workbench, constant temperature CO_2_ incubator (Thermo Scientific); inverted microscope (Olympus); low-temperature ultrahigh speed centrifuge (MCE); low-temperature automatic balancing centrifuge (Beijing Medical Centrifuge Factory); electric thermostatic water tank (Shanghai Medical Instrument Factory No.7); and ultraviolet projection analyzer (Shanghai Yiheng Technology Co., Ltd.) are the main instruments.

## 3. Experimental Method

### 3.1. Cell Culture and Identification

The cell culture method was described previously [1]. Briefly, place the cells in a constant-temperature CO_2_ incubator for 2-4 hours, remove an appropriate amount of the original medium, and gradually mix the old and new medium from less to more during the passage. After the cells are digested, add L-DMEM complete medium (containing 10% fetal bovine serum, 1% streptomycin, 1% cephalosporin, 20 *μ*g/L vascular endothelial growth factor, 2 *μ*g/L insulin-like growth factor 1, 2 *μ*g/L basic fibroblast growth factor, and 20 *μ*g/L epidermal growth factor), the cells are placed in a culture flask with a bottom area of 25 cm^2^ and incubated in a 37°C incubator. The culture medium is replaced every other day, and the proliferation of fibroblasts needs to be replaced every day. When the cell fusion covers more than 90%, the cells are digested with 0.25% trypsin and 0.01% EDTA and cultured at a ratio of 1 : 2. The proliferation rate of the fourth generation human adipose stem cells at the fourth week, the fifth generation human fibroblasts at the third week, and the fifth generation human vascular endothelial cells at the third week was relatively stable. Observe the morphological changes and proliferation of each cell under an inverted phase-contrast microscope.

In the identification of cell surface markers, an immunofluorescence method was used to detect the expression of antibodies against CD90, CD105, CD133, vWF, vimentin, and actin in adherent cells [4]. The cells were planted on 96-well plates, with 5 wells of human adipocyte stem cells and human vascular endothelial cells, 4 of which were stained with fluorescent markers and 1 was used as a negative control group. The samples were washed twice with PBS, fixed with 40 g/L paraformaldehyde for 30 min, dried for 10 min, and incubated with 3% serum albumin for 20 min. Different primary antibodies were added at -4°C and then left to rest overnight, washed with PBS for 3 times. An appropriate amount of sheep anti-rabbit or anti-mouse CY3 fluorescein labeled secondary antibody was added, incubated in a wet box at 37°C for 30 min, washed with PBS for 3 times, soaked with DAPI for 60 s, sealed with 50% buffer glycerol, and observed under a fluorescence microscope.

### 3.2. Experimental Groups and Microscopic Observation

Adipose stem cells, vascular endothelial cells, and fibroblasts were cocultured and divided into the following four groups: (1) adipose stem cell group, (2) adipose stem cell+vascular endothelial cell coculture group, (3) adipose stem cell+fibroblast coculture group, and ④ adipose stem cell+vascular endothelial cell+fibroblast coculture group. Adipose stem cells were placed in 20 6-well plates, and a noncontact coculture model was established through Transwel cells with a pore size of 0.4 *μ*m [5]. The cells were cultured in a 37°C CO_2_ incubator with a volume fraction of 5%. The adipose stem cells in the lower chamber were digested and subcultured every two or three days and cocultured for two weeks under normal conditions and observed and recorded under a microscope. The culture model is shown in Figure 1.

### 3.3. CCK-8 to Detect the Proliferation of Each Group and Plot the Growth Curve

Adipose stem cells of each group cocultured at 1, 3, 5, 7, and 9 days in Step 1.4.2 were taken, and the cell concentration was adjusted to 2 × 10^4^/mL. The cells were inoculated with 100 *μ*L/well in 5 96-well plates, and 4 multiple wells were set in each group of plates. CCK-8 reagent was added to the plates with 10 *μ*L/well. The cells were incubated in the cell incubator for 2 h. Plot the cell growth curve.

### 3.4. Alizarin Red and Alkaline Phosphatase Staining

1. Saturated alizarin red staining: each group of adipose stem cells cocultured at 7, 14, 21, and 28 days in Step 1.4.2 was stained with saturated alizarin red calcium; cells from 1 well of each group were washed with PBS for two or three times and air-dried. An appropriate amount of 10% neutral formaldehyde was added, fixed for 30 min at room temperature, and washed with ultrapure water for two or three times. 0.5% alizarin red staining solution was added, and the staining solution was gently shaken on the shaking table for 5-10 min. PBS was washed once for 15 min, PBS was sucked, and ultrapure water was added, and bone calcium secretion of cells in each group was observed under an inverted microscope.
2. Alkaline phosphatase staining: an azo coupling method was used to measure alkaline phosphatase activity; each group of adipose stem cells cocultured for 7, 14, 21, and 28 days in Step 1.4.2 was used for alkaline phosphatase staining; cells from 1 well in each group were rinsed twice with PBS, then dried, fixed with 40 g/L paraformaldehyde for 30 min, rinsed with distilled water, and added with incubation solution (naphthol As-Bi phosphate 20 mg, dimethyl sulfoxide 0.5 mL, 0.2 mol/L Barbiturate acetic acid buffer 50 mL, hexazo parafuchsin 0.5 mL, and pH 9-10), incubated at room temperature for 45 min, washed with water, and dried. Alkaline phosphatase staining of mixed cells was observed under an inverted microscope.

### 3.5. Western Blot Was Used to Detect the Expression of Bone Morphogenetic Protein 2

Adipose stem cells cultured on day 21 of each group were added into RIPA lysis solution for ice lysis for protein extraction [6], protein concentration was measured by BCA method, SDS-PAGE glue was prepared, protein samples were loaded for separation and membrane transfer and sealed at room temperature with 3% BSA for 1 h, the blocking solution was removed, and PVDF membrane was washed with TBST2. The antibody was incubated in a room temperature shaker for 1 h, and the chemiluminescence was displayed. The relative protein expression level was indicated by the ratio of the gray value of the target band to that of the *β*-actin band [7].

### 3.6. Main Outcome Measures

(1) After 2 weeks of cell culture, the morphology of adipose stem cells was observed under a microscope. (2) CCK-8 was used to detect cell proliferation in each group. (3) The results of saturated alizarin red and alkaline phosphatase staining of adipose stem cells in each group are shown. (4) The expression of bone morphogenetic protein 2, an osteogenic marker of adipose stem cells, was detected by Western blot to evaluate the osteogenic differentiation ability of the coculture system.

### 3.7. Statistical Analysis

All experimental data were expressed as $\bar{\chi \;}\pm s$, with *a* = 0.05 as the test level. One-way ANOVA was used for comparison between groups, a *q* test was used for pair comparison, and statistical software SPSS 26.0 was used for statistical analysis. *P* < 0.05 was considered statistically significant.

## 4. Results

### 4.1. Cell Culture and Identification

#### 4.1.1. Morphological Observation and Identification of Adipose Stem Cells

1. Observed under inverted phase contrast microscope, a large number of spindle cells and polyhedral cells were observed after stable propagation to 4 weeks and 3 generations. The cell body was large, the nucleus was centered, and the growth was in the shape of nests, arranged in a compact and regular way. Surface antigen identification showed that CD90 and CD105 staining of the third generation adipose stem cells were positive in immunofluorescence detection [8], CD133 and vWF were negative, and no positive cells were found in negative control. After 14 days of osteogenesis induction, alkaline phosphatase staining showed that most of the cells were positive, and the cells fused into groups, and the blue and black granules fused with each other and arranged in a network. Alizarine red calcium staining shows partial fusion of cells, forming patchy calcifications with large red nodules of calcium. Staining results proved that the cells had osteogenic differentiation ability, so the obtained cells were determined to be adipose stem cells [9], as shown in Figure 2

(2) In morphological observation and identification of vascular endothelial cells, observed under an inverted phase contrast microscope, the number of cell growth was large and the morphology was diversified, including fusiform and polygon mixed growth, arranged in clumps and bundles, and single scattered distribution. Surface antigen identification showed that CD133 and vWF staining were positive in the immunofluorescence detection of vascular endothelial cells after 3 weeks of subculture [10], CD90 staining was negative, and no positive cells were found in the negative control, as shown in Figure 3

(3) In morphological observation and identification of fibroblasts, the inverted phase contrast microscope showed that there were a large number of cells with large cell bodies, most of which were fusiform and fusiform flat cells but some of which were irregular in shape. The cells were cross-linked with each other by elongated processes and densely arranged in vortex shape. Surface antigen identification showed that vimentin (vimentin) staining was positive and actin (actin) staining was negative in fibroblasts after 3 weeks of subculture [11], and no positive cells were found in negative control, as shown in Figure 4

### 4.2. Cell Morphology Observation

After 2 weeks of cell culture, cell morphology was observed under a microscope, as shown in Figure 5. (1) In the adipose stem cell group, it is single fusiform, without cell overlap. (2) In the coculture group of adipocytes+vascular endothelial cells, the number of cells increased, the cells grew in a vortex shape, and the morphology was diversified, with spindle and polygonal mixed growth. Spindle was more common, and a few were distributed in a nest shape. (3) In the adipose stem cell+fibroblast coculture group, the cell morphology was still simple, showing a long spindle shape and uniform arrangement, and the cell body was larger than average, and there was no cell fusion mass. (4) In the coculture group of adipose stem cell+vascular endothelial cell+fibroblasts, the number of cells increased gradually, most of the cells lost spindle shape, the shape became large and polygonal, and some cells fused into clumps and distributed like nests.

### 4.3. Growth Curve

The absorbance value of adipose stem cells in each group was measured by CCK-8, and the growth curve was drawn. The cell growth curve of each group was similar, and the absorbance value increased gradually. Statistical one-way ANOVA was used for comparison between groups, and a *q* test was used for pairwise comparison of absorbance values in each group. There was no statistical significance in the differences among the groups on day 1 (*P* > 0.05), while pairwise comparison among other groups had significant significance (*P* < 0.05). On day 3, there was no significant difference between the adipose stem cell group and adipose stem cell+fibroblast coculture group (*P* < 0.05). On days 3, 5, 7, and 9, the OD value of adipose stem cell+vascular endothelial cell+fibroblast coculture group was significantly higher than that of the other three groups, and the OD value of adipose stem cell+vascular endothelial cell coculture group was higher than that of adipose stem cell+fibroblast coculture group, with statistical significance (*P* < 0.05), as shown in Figure 6.

### 4.4. Results of Alizarin Red and Alkaline Phosphatase Staining

1. Alizarin red staining analysis of cells in each group: on day 7, cells in each group showed negative reaction. On day 14, a very small number of red positive cells appeared in the mixed culture groups. On day 21, the number of red positive cells increased in the mixed culture group, especially in the coculture group of adipose stem cells+vascular endothelial cells+fibroblasts. On day 28, all cells in each group had red positive cells, and the adipose stem cell+vascular endothelial cell+fibroblast coculture group had the most red focal, while the adipose stem cell+vascular endothelial cell coculture group and adipose stem cell+fibroblast coculture group were less and the adipose stem cell group was the least, as shown in Figure 7.

(2) Alkaline phosphatase staining analysis of cells in each group: on day 7, positive particles appeared in all groups except the adipose stem cell group, and the most positive particles appeared in the adipose stem cell+vascular endothelial cell+fibroblast coculture group. On day 14, red positive particles appeared in all groups, which were more obvious in adipose stem cell+fibroblast coculture group and adipose stem cell+vascular endothelial cells+fibroblast coculture group. On day 21, the number of red positive particles increased in the mixed culture group, especially in the coculture group of adipose stem cells+vascular endothelial cells+fibroblasts. On day 28, with the exception of adipose stem cell group which is not obvious, the rest of the groups of cells have obvious positive particles, red fat stem cell+fibroblast trained group, the fat cells, vascular endothelial cell and fibroblast trained group, the most fat stem cell+endothelial cell coculture group, and adipose stem cell group, as shown in Figure 8

### 4.5. Western Blot to Detect the Expression of Bone Morphogenetic Protein 2

Bone morphogenetic protein 2 was expressed in adipose stem cells of each group and was more obvious in the adipose stem cell+fibroblast coculture group and adipose stem cell+vascular endothelial cell+fibroblast coculture group, as shown in Figure 9. There was no statistically significant difference between the adipose stem cell group and the adipose stem cell+vascular endothelial cell coculture group (*P* > 0.05), while there was statistically significant difference between the other groups (*P* < 0.05), as shown in Figure 10.

## 5. Discussion

Tissue engineering includes three key factors, tissue materials, and growth factors. As one of the highlights of scientific research in China's agricultural sciences, the ideal cell product should have good biological functions such as cell activity, plant, production, and synthesis [12]; the properties of mesenchymal stem cells with multidirectional bands and characteristics have been extensively studied [12]. Although mesenchymal stem cells are mostly distributed in bone marrow and cord blood, they are very low in peripheral blood and have inhibitory effects [13]. When grown up, fibroblasts exist in various tissues of the body and can be obtained easily and quickly. They can be autologously transplanted and can be huge [3]. The mesenchyme is also phenotypic. They are similar in cell morphology and development, and fibroblasts have cell characteristics that they do not have: bone cells, osteocalcin, bone morphogenetic protein, type II material particles, and phosphatase-free expression of osteoblast markers [2]. Therefore, fibroblasts have gradually become the preferred seed cell model for tissue research.

The coculture of fibroblasts and stem cells can promote stem cell proliferation and induce differentiation by secreting fibroblast factors and participating in MAPK-mediated signaling pathways [14]. In recent years, fibroblast growth factor is considered to play a key role in the growth and development of the skeletal system and fracture healing [15]. At least 23 related factors have been found, including fibroblast growth factor 2, fibroblast growth factor 8, fibroblast growth factor 18, and fibroblast growth factor 21. Fibroblast growth factor binds to the fibroblast growth factor receptor on the cell surface to induce the receptor to activate cell signaling pathways such as erK1/2 and JNK, regulate target gene transcription, and promote osteogenic differentiation. In vitro and in vivo studies have confirmed that fibroblast growth factor 2 can also promote cell osteogenesis by promoting *β*-catenin expression and nuclear accumulation [16]. Different types of fibroblast growth factors have different effects on different cells. Signal pathways such as ERK and JNK are also involved in the interaction of fibroblast growth factors and bone morphogenetic proteins, which have an impact on osteogenesis [17]. In this study, fibroblasts were selected as seed cells, and the coculture system confirmed that they have a certain osteoinductive effect on adipose stem cells. In this study, osteocalcin and bone morphogenetic protein were used to evaluate bone formation performance. Osteocalcin is the most characteristic secretion of osteoblasts, and its appearance can directly mark the maturation of osteoblasts and is recognized as a characteristic phenotype of advanced osteoblast differentiation [18]. Western blot can be used to detect the expression of bone morphogenetic protein 2 [19]. Bone morphogenetic protein 2 (BMP 2) is a bone formation promoter and a member of the transforming growth factor beta superfamily [20]. Bone morphogenetic protein 2 can promote the expression of osteocalcin and alkaline phosphatase and promote the synthesis of osteopontin, osteocalcin, and type I collagen and the mineralization of extracellular matrix [21, 22], thereby promoting osteoblasts and the maturation, proliferation, and differentiation of osteoblasts and induces new bone formation in vivo and in vitro [23].

In recent years, the construction of single-cell tissue engineering can no longer meet the requirements of simulating tissue structure and physiological effects, maintaining tissue stability and vitality [24]. Especially in the absence of vascular tissue construction, a good blood supply is the key to the success of tissue engineering treatment [25]. Not only a good blood supply is required, but also the presence of diverse cellular components [26]. More and more researchers tend to use multicell culture to build seed cell systems [6]. When studying the multicell coculture system, direct and indirect coculture methods used in tissue engineering, and the characteristics of the interaction of various cells in coculture, it is proposed that the coculture system is controlled by the interaction of various cell types and signal transduction cell behavior [27]. In the coculture system of fibroblasts, vascular endothelial cells, and adipose stem cells, the cytokines secreted by fibroblasts and vascular endothelial cells interact to promote the proliferation and osteogenic differentiation of adipose stem cells [28]. The crosstalk between vascular endothelial growth factor and bone morphogenetic protein 6 signaling pathway enhances the osteogenic differentiation of mesenchymal stem cells [29]. The coculture of extracellular matrix and fibroblasts has a higher potential to promote the differentiation of mesenchymal stem cells into vascular smooth muscle cells [30]. Rat bone marrow mesenchymal stem cell membranes show high osteogenic differentiation potential under the induction of basic fibroblast growth factor and can increase the expression level of transforming growth factor *β*1 in the late stage of osteogenesis [31]. The three-dimensional coculture of BMSCS transfected with basic fibroblast growth factor and ligament fibroblasts can promote the proliferation of BMSCS and enhance its ability to differentiate into ligament fibroblasts. Previous studies have confirmed that the combined culture of vascular endothelial cells and adipose stem cells can effectively promote the proliferation and osteogenic differentiation of adipose stem cells [32]. However, normal bone tissue contains a large number of fibroblasts, which have excellent proliferation and differentiation properties, collagen secretion, and synthesis capabilities and contain a variety of regulatory fibroblast growth factors [33]. In the coculture system, the cytokines secreted by vascular endothelial cells and fibroblasts can provide a microenvironment for the proliferation and differentiation of adipose stem cells, because of the joint action of bone morphogenetic protein-2, vascular endothelial growth factor, and fibroblast growth factor, promoting the generation and differentiation of osteoblasts [34–37]. This study established a coculture system of fibroblasts, adipose stem cells, and vascular endothelial cells and found that the coculture of the three has a certain effect on the proliferation and osteogenic differentiation of adipocytes.

## 6. Conclusion

In conclusion, the adipose stem cell+vascular endothelial cells+fibroblast coculture group had the strongest ability to promote the proliferation of adipose stem cells and differentiate into osteoblasts rapidly and efficiently. The coculture of adipose stem cells with vascular endothelial cells and fibroblasts has great research potential. In the next research, it can be considered to provide seed cells for tissue engineering and provide a new idea for tissue engineering to construct biological scaffolds for repairing bone defects. However, the factors affecting cell proliferation and differentiation in the coculture system and the regulatory mechanism are not clear at present, so the interaction factors of the three kinds of cells in the coculture system can be studied in the future.

## Figures and Tables

**Figure 1:** Cell culture model. (a) is ADSCs cultured alone; (b) was ADSC+VEC coculture (VECs was located in the upper compartment and ADSCs in the lower compartment); (c) was ADSC+FB coculture (FB was located in the upper compartment and ADSCs in the lower compartment); (d) was ADSC+VEC+FB coculture (VECs and FB were located in the upper compartment by the direct contact coculture method, and ADSCs were located in the lower compartment). ADSCs: adipose stem cells; VECs: vascular endothelial cells; FB: fibroblasts.

**Figure 2:** Morphology, immunofluorescence staining, and osteogenic induction identification of adipose stem cells. (a) and (b) are adipose stem cells with magnification of 100 and 40 times, respectively (inverted phase contrast microscope). (c) is CD90 staining (fluorescence microscope, ×100); (d) is CD105 staining (fluorescence microscope, ×100); (e) is CD133 staining (fluorescence microscope, ×100); (f) is vWF staining (fluorescence microscope, ×100); (g) is alkaline phosphatase staining (fluorescence microscope, ×100); (h) is alizarin red calcium staining (fluorescence microscope, ×100) ((a, g, h) scale of 50 *μ*m, (b) scale of 100 *μ*m, and (c–f) scale of 200 *μ*m).

**Figure 3:** Morphological observation and immunofluorescence staining identification of vascular endothelial cells. (a) and (b) are vascular endothelial cells with magnification of 100 and 40 times, respectively (inverted phase contrast microscope). (c) is CD133 staining (fluorescence microscope, ×100); (d) is vWF staining (fluorescence microscope, ×100); (e) is CD90 staining (fluorescence microscope, ×100) ((a) scale of 50 *μ*m, (b) scale of 100 *μ*m, and (c–e) scale of 200 *μ*m).

**Figure 4:** Morphological observation and immunofluorescence staining identification of fibroblasts. (a) and (b) are fibroblasts with magnification of 100 and 40 times, respectively (inverted phase contrast microscope). (c) is for vimentin staining (fluorescence microscope, ×100); (d) is actin staining (fluorescence microscope, ×100) ((a) scale of 50 *μ*m, (b) scale of 100 *μ*m, and (c, d) scale of 200 *μ*m).

**Figure 5:** Morphological observation of adipose stem cells in each group (×100, scale: 50 *μ*m). (a)–(d) are the ADSC group, ADSC+VEC group, ADSC+FB group, and ADSC+VEC+FB group, respectively. ADSCs: adipose stem cells; VECs: vascular endothelial cells; FB: fibroblasts.

**Figure 6:** Growth curves of adipose stem cells cultured in each group. There was no statistically significant difference between each group on day 1 (*P* > 0.05), and there was no statistically significant difference between the adipose stem cell group and adipose stem cell+fibroblast coculture group on day 3 (*P* < 0.05). On days 3, 5, 7, and 9, the OD value of adipose stem cell+vascular endothelial cell+fibroblast coculture group was significantly higher than that of the other three groups, and the OD value of adipose stem cell+vascular endothelial cell coculture group was higher than that of adipose stem cell+fibroblast coculture group, with statistical significance (*P* < 0.05).

**Figure 7:** Alizarin red staining of adipose stem cells at each time point of coculture (scale: 50 *μ*m). (a–d) In the figure are the ADSC group, ADSC+VEC group, ADSC+FB group, and ADSC+VEC+FB group, respectively. On day 28, there were red positive cells in all groups, and the ADSC+VEC+FB group was the most and ADSC group was the least. ADSCs: adipose stem cells; VECs: vascular endothelial cells; FB: fibroblasts.

**Figure 8:** Alkaline phosphatase staining of adipose stem cells at each time point of coculture (scale: 50 *μ*m). (a–d) In the figure are the ADSC group, ADSC+VEC group, ADSC+FB group, and ADSC+VEC+FB group, respectively. On day 28, except the adipose stem cell group, cells in other groups had obvious red positive particles. The adipose stem cell+fibroblast coculture group and adipose stem cell+vascular endothelial cell+fibroblast coculture group had the most, and adipose stem cell+vascular endothelial cell coculture group had less. ADSCs: adipose stem cells; VECs: vascular endothelial cells; FB: fibroblasts.

**Figure 9:** Expression of BMP-2 detected by Western blot.

**Figure 10:** The expression of bone morphogenetic protein 2 in adipose stem cells. ADSCs: adipose stem cells; VECs: vascular endothelial cells; FB: fibroblasts. At the same time point, compared with ADSCs, ^a^*P* < 0.05; compared with ADSCs+VECs, ^b^*P* < 0.05; compared with ADSCs+FB, ^c^*P* < 0.05.

## Data Availability

The data used to support the findings of this study are included within the article.
